The article "Relationship between Economic Growth and Energy Consumption from the Perspective of Sustainable Development" was retracted in 2023. Reasons: unreliable results or conclusions; concerns about the data; concerns about the results or conclusions; concerns about the peer review.

# Relationship between Economic Growth and Energy Consumption from the Perspective of Sustainable Development

**DOI:** 10.1155/2022/6884273

**Published:** 2022-07-20

**Authors:** Liuyi Dai, Rui Jia, Xinran Wang

**Affiliations:** ^1^Department of Economics, Pusan National University, Busan 46241, Republic of Korea; ^2^Baotou Teachers' College, Inner Mongolia University of Science and Technology, Baotou 014030, Inner Mongolia, China; ^3^Department of Business Administration, Pusan National University, Busan 46241, Republic of Korea; ^4^Department of Business Administration, Jeonju University, Jeonju 55069, Republic of Korea

## Abstract

While promoting the economic growth, energy has also brought pollution problems to the world environment, which has gradually become a bottleneck impeding sustainable economic development. In view of the rapid evolution of urbanization and industrialization, economic growth is increasingly dependent on the energy consumption, the development of the two is difficult to coordinate, and the internal contradictions are becoming increasingly serious, which hinders the sustainable development of economic growth. This study establishes the relationship between energy consumption and economic growth according to the energy Kuznets curve and studies the future trend of China's sustainable development through the comparative analysis of the energy Kuznets curve of the United States and Germany. The results show that, at the turning point of energy consumption, China's energy economic rate is higher than that of Germany and the United States. In addition, in terms of urbanization rate and industrial structure, although China's tertiary industry has made a breakthrough, it is still lower than that of the United States and Germany, but the level of urbanization rate has made significant progress. In short, China has obvious advantages in future economic development and has a late developing advantage compared with the United States and Germany. This paper makes an empirical analysis of the relationship between energy consumption and economic growth in OECD countries and finds out the turning point of energy consumption, so as to provide a theoretical basis for coordinating China's energy consumption and economic growth.

## 1. Introduction

As an important material basis for the development of human society, energy is also the main driving force of economic growth. However, while energy promotes the economic growth, it also brings pollution problems to the world environment and gradually becomes the bottleneck hindering the sustainable development of the economy [1]. In view of the fact that the pace of China's modernization and urbanization is intensifying, environmental pollution has become the main problem restricting China's economic development, and the demand for energy consumption continues to increase. In view of this, realizing the coordinated development of energy consumption and economic growth and clarifying the future economic development direction of China are the main breakthroughs in building a moderately prosperous society in an all-round way [2]. In view of the Kuznets curve of energy consumption and economic growth, the contradiction between energy consumption and economic growth has become an important breakthrough direction to achieve sustainable economic development [3]. Therefore, to overcome the inherent contradiction between economic growth and energy consumption and realize the coordinated development of the two is the only way for China to solve the future economic development plan and establish a sustainable economic development path [4].

Analyzing the relationship between energy and economic development from the perspective of economics, there are mainly two aspects, first, the economic development is dependent on energy. That is, the economic development is inseparable from energy. Secondly, the degree and scale of energy opening and utilization are based on certain economic development conditions. Economic development can promote the large-scale development and utilization of energy. In order to explore the internal relationship between China's energy consumption and economic growth, economists use a large number of measurement methods to study the statistical data from different periods. The data show that the results are very different. Energy is introduced into the Cobb Douglas production function as a new variable. A VAR model is established, and a conclusion is drawn that China's energy consumption is related to the economic growth. Because the relationship between China's power consumption and China's energy consumption and economic growth is in a complex economic system, any different initial or research methods may lead to completely different results.

In view of the relationship between energy consumption and economic growth, this study describes the energy Kuznets curve, establishes the economic turning point of energy consumption, explores the regularity of economic growth and energy consumption, and excavates the economic planning and development strategy suitable for China's sustainable development road by drawing the energy Kuznets curve and establishing the economic turning point of energy consumption. Then, by forecasting the historical data of China's energy consumption and economic growth, we find out the future turning point of China's energy consumption and finally provide strategic experience for coordinating China's energy consumption and economic growth.

The innovation of this study is that, in order to determine the inherent law of economic growth and energy consumption and to overcome the contradiction between them in the development process, this paper empirically analyzes the relationship between energy consumption and economic growth in OECD (Organization for Economic Co-operation and Development) countries and finds out the turning point of energy consumption, so as to provide a theoretical basis for coordinating China's energy consumption and economic growth. After that, it evaluates the relevant data of China's energy consumption and economic growth, constructs the energy Kuznets curve, and establishes the turning point of China's energy development in the future, and through the comparative analysis of the relevant data of the United States and Germany, the specific similarities and differences are analyzed so as to provide practical experience for promoting the road of sustainable development in China.

The main structure of the paper is divided into four parts. Firstly, the paper compares and analyzes the Kuznets curve of energy between the United States and Germany, finds out the essence of the energy turning point law, analyzes the regular content between the energy consumption and economic growth in the United States and Germany with reference to the historical data, and subdivides the relationship between the urbanization rate, industrial structure, and other related factors and the energy turning point. Secondly, it analyzes the relationship between energy consumption and economic growth in China, establishes the energy turning point, and makes a comparative analysis with the United States and Germany. Finally, according to the relationship between China's economic growth and energy consumption, we should make clear the direction of China's economic development and promote the road of sustainable development in China.

## 2. Related Work

Pla Julian and Guevara pointed out that, for the economic development based on sacrificing the natural ecological environment, the goal and consensus of sustainable development should be established to ensure the sustainable development of the Earth. Transforming consumption and the production processes is a fundamental priority of this development agenda. As an alternative model, the circular economy has emerged because of its potential to create a value and has positive social and environmental impacts (Pla Julian and Guevara) [5]. Eihigiamusoe and Lean used the first and the second-generation cointegration and estimation procedures to solve the different economic and econometric problems and found that there is a cointegration relationship between the variables. In the whole sample, energy consumption, economic growth and financial development have adverse effects on the carbon emissions, and energy consumption will increase the carbon emissions. The results show that the high-income level and financial development can reduce the carbon emissions, while low-income and financial development may aggravate the carbon emissions (Ehhigiamusoe and Lean) [6]. The results show that energy consumption has a positive and a significant impact on the economic growth. There is a positive correlation between the financial development and economic growth (Sadraoui et al.) [7]. According to the nonstationary time series that may appear in some provinces, the autoregressive distribution lag (ARDL) modeling method is adopted. The estimation results show that the relationship between per capita energy consumption and per capita GDP varies greatly among provinces [8]. Asumadu and Vladimir used panel data regression with the Driscoll Kraay standard error and the *U* test estimation method and panel quantile regression with the nonadditive fixed effect. It is found that the energy consumption has a strong positive impact on the greenhouse gas emissions (Asumadu and Vladimir) [9]. Jin and Yu pointed out that the China's total energy consumption has increased sharply, and also China's dependence on coal is relatively high. This has also brought about serious environmental problems, which will become one of the main reasons for restricting China's economic development (Jin and Yu) [10].

Using the annual data from 1980 to 2011, Deonanan and Ramkissoon studied the causal relationship between energy consumption and economic development in 13 Caribbean small island developing states. The multivariate model including the environmental emissions is estimated, and the Granger causality is tested by the Toda-Yamamoto method to determine the causality of each country. The evidence for the four different types of causality was found. These results have an impact on the various energy policies in the Caribbean economies (Deonanan and Ramkissoon) [11]. Tran et al used the system generalized moment method (SGMM) to comprehensively estimate the three simultaneous equations of human development, energy consumption, and dioxin emissions in 90 countries from 1990 to 2014. The results showed that the improvement of human development level leads to the reduction of carbon emissions in global sample countries and developing countries. However, in developed countries, there is no significant relationship between the carbon emissions and human development (Tran et al) [12]. Mohsin et al. used the econometric method to test the relationship between economic growth and energy consumption. The research results showed that economic growth at the cost of energy consumption leads to urban environmental degradation, and it is difficult to carry out the sustainable development path (Mohsin et al) [13]. Erzi et al established a model based on the heterogeneous productivity to analyze the macroeconomic problem of energy consumption changing with the economic development when the economy becomes more productive. Studies have shown that when an economy becomes more productive, it will have more output and will input more resources, and most importantly, energy will also increase (Erzi et al ) [14]. Taking nine resource-based regions in China as the research objects, Hao and Deng used the variable coefficient panel model and the Hansen panel threshold model to quantify the marginal effect and threshold effect of innovation ability in optimizing energy consumption structure. The results show that the total index of energy consumption structure in the analysis region is 0.563, indicating that the structure is relatively low, and the regional economic development mainly depends on low-grade energy (Hao and Deng) [15].

Through the relevant research on economic growth and energy consumption by many scholars at home and abroad, we can see that the regular content between the energy consumption and economic growth is analyzed, and the relationship between the urbanization rate, industrial structure, and other related factors and the energy turning point is subdivided [16]. To analyze the relationship between energy consumption and economic growth in China, it is very important to establish the energy turning point. In short, the relevant literature shows the theoretical analysis of the relationship between energy consumption and economic growth, establishes the inherent law between the two and the empirical analysis of the relationship between the energy consumption and economic growth in various countries, and finds out the turning point of energy consumption is an important theoretical basis for coordinating energy consumption and economic growth [17].

## 3. Empirical Analysis of Economic Development and Energy Consumption in OECD Countries

### 3.1. Analysis of US Energy Kuznets Curve

In view of the relationship between energy consumption and economic growth, this study describes the energy Kuznets curve, establishes the economic turning point of energy consumption, explores the regularity of economic growth and energy consumption, and excavates the economic planning and economic development suitable for China's sustainable development. Then, by forecasting the historical data of China's energy consumption and economic growth [18], we find the future turning point of China's energy consumption, and finally, it provides a strategic experience for coordinating China's energy consumption and economic growth. In view of this, this study first verifies whether there is an “inverted U” relationship between the economic growth and energy consumption in OECD countries, and then through the identification of their internal regularity and the turning point of energy consumption, the contradiction between energy consumption and economic growth can be overcome. In order to directly reflect the turning point of energy consumption [19], this study selects Germany, the United States, Australia, Canada, and the United Kingdom as the research objects and analyzes the relationship between energy consumption and economic growth of these five countries as a whole and draws up the “inverted U” curve of these five countries, as shown in Figure 1.

As can be seen from Figure 1, with the increase in per capita GDP, per capita energy consumption decreased significantly. For Germany, there will be a turning point in the trend when the per capita GDP reaches its peak. Compared with the other three countries, the per capita energy consumption of the UK and Germany is relatively stable. However, for Canada and Australia, their energy consumption fluctuates greatly, which shows that there is a significant relationship between the economic growth and energy consumption. For the United States, the per capita GDP corresponding to its energy consumption is the highest. The reason why the relationship between energy consumption and economic growth in the five countries is quite different is mainly due to the different industrial structures and economic policies of specific countries, which leads to the great difference between energy consumption and economic growth [20]. According to Figure 1, when compared with other countries, Germany has the first energy consumption turning point, followed by the United States and the United Kingdom, and Canada has a late energy consumption turning point. It was not until 2006 that Australia saw a turning point in energy consumption. In order to further analyze the relationship between energy consumption and economic growth, we explore the regularity of economic growth and energy consumption and dig out the economic planning and economic development suitable for China's sustainable development. This study also analyzes the relationship between the urbanization rate, industrial structure, per capita GDP, and energy consumption, so as to find out the important factors that affect the turning point of energy consumption. The specific results are shown in Table 1.

From Table 1, it can be concluded that the United States, Germany, the United Kingdom, and Canada reached the turning point of energy consumption in 2000. Therefore, energy consumption is an important prerequisite for economic growth. The turning point of energy consumption corresponding to unit GDP energy consumption is relatively low. The improvement of technical level can effectively improve the energy consumption rate, that is, the improvement of technical level can strengthen the utilization rate of energy. In addition, the optimization of industrial structure can accelerate the emergence of energy consumption turning point. At the same time, the urbanization rate can also promote the emergence of the energy consumption turning point. In short, through the analysis of the relationship between energy consumption and economic growth in the United States, Germany, the United Kingdom, Canada, and Australia, the “inverted U” curve shows that there is a positive correlation between the economic growth and energy consumption, that is, the greater the energy consumption, the faster the economic growth. However, when the economy grows to a certain level, the government's attention to energy issues, the improvement of technical level, the optimization of industrial structure, and the innovation of the economic system are of great importance to the improvement of energy utilization rate, and the turning point of energy consumption appears.

### 3.2. Analysis of the US Energy Kuznets Curve

In the face of the relationship between energy consumption and economic growth, the US energy policy is quite typical. The state improves the utilization rate of energy consumption by formulating corresponding policies and statistical innovation, that is, coordinating the relationship between energy production and distribution and economic growth. It can be said that the United States has a comprehensive strategic plan and vision at the level of energy policy. Among them, the United States has formulated three energy policy principles, namely, the principle of a long-term comprehensive strategy, the principle of coordinated development between clean and efficient development and environmental and ecological construction, and the principle of an effective combination of per capita living standard construction and energy and environmental policies. Specifically, the industrial structure and urbanization rate of the United States are shown in Figure 2.

The primary industry refers to the industries that produce aquatic, native, and agricultural raw products, such as agriculture, forestry, and fishing. The secondary industry refers to the industries that process the raw materials of the primary industry and this industry. The common ones are mining, manufacturing, construction, and so on. The tertiary industry refers to the industries other than the primary industry and the secondary industry that are independent. The common ones are transportation, catering, real estate, and so on. It can be seen from Figure 2 that, historically, the energy consumption in the United States is mainly wood energy. After that, energy consumption has shifted from wood to coal and then from coal to oil. Until the second half of the last century, energy consumption in the United States was mainly coal, oil, and natural gas, accounting for more than 80%. With the development of the economy and technology in the United States, renewable energy appears in the energy structure of the United States, and the sustainable utilization of the renewable energy effectively reduces the consumption of coal, natural gas, and oil. It can be said that the technological innovation has gradually turned the energy consumption of the United States to renewable energy and directly coordinated the relationship between the traditional energy consumption and economic growth. The changing trend of energy consumption structure and energy consumption per unit of GDP in the United States is shown in Figure 3.

According to the relevant data from the world bank, this paper compares the growth rate of per capita GDP and the growth rate of energy consumption in the United States since 1961. The results show that, with the growth or recession of the US economy, the energy consumption basically remains unchanged. In addition, the regression analysis shows that the relationship between economic growth and energy consumption is inverted U-shaped. In order to find the turning point more intuitively, the relationship between per capita energy consumption and per capita GDP in the United States is fitted into an inverted U-shaped curve. On the whole, the US economic growth and energy consumption “inverted U” curve has high stability and does not have large fluctuations. Among them, the US per capita energy consumption and per capita GDP growth rate and its “inverted U” curve are shown in Figure 4.

By analyzing the relationship between the economic growth and energy consumption in the United States, it is seen that the energy consumption is the main driving force to promote economic growth. However, while energy promotes the economic growth, it also brings pollution problems to the world environment, and it gradually becomes the main problem hindering the sustainable development of the economy. This study, through determining the inherent law of economic growth and energy consumption, it finds out the turning point of energy consumption and then overcomes the internal contradiction between energy consumption and economic growth so as to provide the theoretical basis for coordinating energy consumption and economic growth in China. As can be seen from Figure 4, with the growth or recession of the US economy, the trend of energy consumption remains basically unchanged. In addition, the regression analysis shows that, in the relationship between economic growth and energy consumption, the relationship between per capita energy consumption and per capita GDP in the United States is inverted U-shaped, and the “inverted U” curve between the economic growth and energy consumption in the United States is stable and does not have large fluctuations. On the whole, it is very important to see through the relationship between energy consumption and economic growth in the United States, to explore the regularity of the economic growth and energy consumption and to dig out the economic planning and economic development suitable for China's sustainable development.

### 3.3. Kuznets Curve Analysis of German Energy

By exploring the relationship between energy consumption, urbanization rate, and industrial structure, it is found that the German urbanization rate is relatively stable, but the industrial structure changes greatly. The specific results are shown in Figure 5.

Compared with other countries, Germany's economic situation is mainly characterized by developed industrialization but restricted by its own natural environment, resulting in the shortage of natural resources in Germany. In view of the positive correlation between economic growth and energy consumption, it is difficult for German industry to develop sustainably and healthily. It is necessary to optimize the energy structure and to develop new energy so as to reduce the economic development obstacles caused by its own energy defects. The historical energy consumption structure and unit energy consumption trend of Germany is shown in Figure 6.

It can be seen from Figure 6 that Germany's economic growth is stable, but the energy consumption is not stable. According to the regression analysis of the energy consumption, the relationship between per capita energy consumption and per capita GDP in Germany is fitted into an inverted U-shaped curve. After entering the turning point, Germany's per capita energy consumption shows a significant downward trend. Among them, the Germany's per capita energy consumption and the GDP growth rate and its “inverted U” curve are shown in Figure 7.

In view of the Kuznets curve of energy consumption and economic growth, the contradiction between the energy consumption and economic growth has become an important breakthrough direction to achieve sustainable economic development. Therefore, to explore the coordinated development of the energy consumption, economic growth is the only way to solve the future economic development plan and establish a sustainable economic development path. This study establishes the relationship between energy consumption and economic growth according to the energy Kuznets curve and studies the future trend of China's sustainable development by comparing and analyzing the energy Kuznets Curves of the United States and Germany.

## 4. Experimental Design and Analysis

### 4.1. Analysis of Kuznets Curve Results of China's Energy

This study establishes the relationship between energy consumption and economic growth according to the energy Kuznets curve and studies the future trend of China's sustainable development by comparing and analyzing the energy Kuznets Curves of the United States and Germany. At a specific level, the turning point of China's energy consumption is predicted and analyzed by analyzing the historical data of the energy consumption and economic growth in China. The methods quadratic equation was used for regression analysis (Table 2).

In order to visualize the relationship between China's energy consumption and economic growth, this study makes an inverted U curve fitting between China's future energy consumption and per capita GDP. Among them, the “inverted U” curve fitting diagram of China's per capita energy consumption and per capita GDP is shown in Figure 8.

It is predicted that China's per capita GDP will reach a turning point of 17138 U.S dollars in the future. According to the above data, China may reach the turning point of energy consumption around the year 2035. At this time, the relevant data on China's economic development and energy consumption are shown in Table 3.

### 4.2. Comparative Analysis of the Kuznets Curves of the Three Countries

Economic development is closely related to energy demand. According to the results of the above analysis, this study studies the future trend of China's sustainable development by comparing and analyzing the Kuznets Curves of the US and Germany. The “inverted U” curve fitting diagram of energy consumption and economic z-growth in the United States, Germany, and China is shown in Figure 9.

According to the prediction, by 2035, China's urbanization and industrialization will become more and more mature. The growth rate of the economic indicators has slowed down significantly, and the proportion of tertiary industry in GDP has increased significantly, which has become the main force driving the economic development. The flow of population to cities tends to slow down, and the growth rate of urbanization gradually slows down. Among them, the economic and energy-related data at the turning point of energy consumption are shown in Table 4.

At the turning point of energy consumption, compared with Germany and the United States, the China's energy economic rate is higher. In addition, in terms of urbanization rate and industrial structure, although China's tertiary industry has made breakthroughs, it is still lower than that of the United States and Germany, but it has made significant progress in the level of urbanization rate. In short, China's economic development in the future has obvious advantages, compared with the United States and Germany, and has the advantages of late development.

## 5. Conclusion

As an important material basis for the development of human society, energy is also the main driving force of economic growth. However, while energy promotes the economic growth, it also brings pollution problems to the world environment and gradually becomes the bottleneck, hindering the sustainable development of the economy. In view of the rapid evolution of urbanization and industrialization, the dependence of the social development on energy consumption continues to increase, leading to the contradiction between economic growth and energy consumption. In view of this, how to coordinate energy consumption and economic growth has become an important breakthrough in sustainable development. This study describes the energy Kuznets curve, establishes the economic turning point of energy consumption, explores the regularity of economic growth and energy consumption, and excavates the economic planning and economic development suitable for the road of sustainable development in China. Then, by forecasting the historical data of China's energy consumption and economic growth, we find out the future turning point of China's energy consumption and finally provide strategic experience for coordinating China's energy consumption and economic growth. The results show that, at the turning point of energy consumption, China's energy economic rate is higher than that of Germany and the United States. In addition, in terms of urbanization rate and industrial structure, although China's tertiary industry has made breakthroughs, it is still lower than that of the United States and Germany, but it has made significant progress in the level of urbanization rate. In addition, it is found that China may have a turning point of energy consumption in 2035, which has a late development advantage compared with the United States and Germany. In view of the fact that China's development is bound to be constrained by high energy consumption, in order to coordinate the development of energy consumption and economic growth, this paper puts forward some suggestions, such as accelerating the strategic adjustment of industrial structure, improving the production and small consumption of energy structure and increasing the proportion of renewable energy consumption. However, there are still some problems in this paper. There is no indepth discussion on the influencing factors of the economic turning point of energy consumption, and further discussion and analysis are needed in the future research.

## Figures and Tables

**Figure 1:** “Inverted U” curve fitting diagram of per capita energy consumption and per capita GDP in different countries.

**Figure 2:** Industrial structure and urbanization rate in the United States. (a) American industrial structure and (b) urbanization rate in the USA.

**Figure 3:** The trend of energy consumption structure change and energy consumption per unit GDP in the United States. (a) Energy consumption structure in the USA and (b) unit energy consumption in the USA.

**Figure 4:** Comparison of per capita energy consumption and GDP growth in the United States and its “inverted U” curve. (a) Comparison of energy consumption and GDP and (b) the “inverted U” curve fitting diagram.

**Figure 5:** The trend of German industrial structure and urbanization rate. (a) Germany industrial structure and (b) urbanization rate in Germany.

**Figure 6:** Historical energy consumption structure and unit energy consumption trend in Germany. (a) Energy consumption structure in Germany and (b) unit energy consumption in Germany.

**Figure 7:** Comparison of per capita energy consumption and GDP growth in Germany and its “inverted U” curve. (a) Comparison of energy consumption and GDP and (b) “inverted U” curve fitting diagram.

**Figure 8:** “Inverted U” curve fitting diagram of China's per capita GDP and per capita energy consumption.

**Figure 9:** U-shaped curve fitting between per capita energy consumption and per capita GDP in the United States, Germany, and China.

**Table 1:** Indicators of economy, energy, and the environment when the energy consumption turning point appears.

Five OECD countries (year)	GDP per capita (USD)	Per capita energy consumption (tons)	Energy consumption per unit GDP (T/10000)	CO_2_ emissions per capita (tons)	Ratio of three industrial structure (%)	Urbanization construction rate (%)
USA (1994)	29249.7	11.1	0.45	19.5	1.8 : 26.2 : 72.0	76.9
Australia (2006)	24310.7	8.0	0.40	17.9	3.1 : 28.0 : 68.9	88.4
Germany (1988)	18144.8	6.6	0.44	—	1.8 : 38.1 : 60.1	72.9
Britain (1994)	20908.1	5.3	0.31	9.6	1.7 : 30.4 : 67.9	78.3
Canada (1999)	22480.9	11.4	0.61	16.8	2.5 : 31.2 : 66.3	79.1

**Table 2:** Regression analysis parameters of China's per capita GDP and per capita energy consumption.

Constant *α*	Parameter *β*2	Parameter *β*2	R2	*F* value	Turning point
623.3669	0.333999	−9.7 E-0.6	0.898025	176.1262	17138.16

**Table 3:** Forecast data of China's economic development and energy consumption in 2035.

Per capita GDP (USD)	Ratio of three industrial structures (%)	Urbanization rate (%)	Per capita energy consumption (kg ce)	GDP energy intensity (ton standard)
17138.2	4.6 : 37.2 : 58.2	72	3800	0.31

**Table 4:** Economic and energy-related data at the turning point of energy consumption.

Country	Index				
	Per capita GDP (USD)	Ratio of three industrial structures (%)	Urbanization rate (%)	Per capita energy consumption (kg ce)	GDP energy intensity (ton standard)
China	17138.2	4.6 : 37.2 : 58.2	72	3800	0.31
USA	29655.1	1.8 : 26.2 : 72.0	76.9	11.1	0.45
Germany	18144.8	1.8 : 38.1 : 60.1	72.9	6.6	0.44

## Data Availability

The data used to support the findings of this study are included within the article.
